# Early Warning Model of Placenta Accreta Spectrum Disorders Complicated with Cervical Implantation: A Single-Center Retrospective Study

**DOI:** 10.1155/2022/8128689

**Published:** 2022-02-04

**Authors:** Siming Xin, Hong Wan, Xiaoming Zeng, Yanyan Fu, Zhizhong Wang, Hua Lai, Ying Xiong, Jiusheng Zheng, Lingzhi Liu

**Affiliations:** ^1^Department of Obstetrics, Maternal and Child Health Hospital Affiliated to Nanchang University, Nanchang 330006, Jiangxi, China; ^2^Department of Preventive Health Care, Maternal and Child Health Hospital Affiliated to Nanchang University, Nanchang 330006, Jiangxi, China

## Abstract

**Background:**

Placenta accreta spectrum (PAS) disorders seriously threaten the safety of the mother and infant in the perinatal period. Moreover, PAS is associated with poor maternal and perinatal outcomes once complicated with cervical implantation. Dismally, there are few reports about PAS complicated with cervical involvement currently, and the early warning models are also rarely reported. To screen the risk factors of PAS complicated with cervical implantation and construct an early risk warning model, we performed the analysis of clinical indicators and images of PAS patients by artificial intelligence (AI) data processing methods.

**Methods:**

The clinical data of 166 patients with PAS in our hospital from January 2016 to September 2020 were retrospectively analyzed. The patients were divided into cervical implantation group and lower uterine implantation group according to the position of placenta implantation. Then, we compared the pregnancy outcomes of the two groups, screened the possible related factors of PAS complicated with cervical implantation by univariate analysis, and established the early warning model by logistic regression analysis.

**Results:**

The maternal outcome of PAS complicated with cervical implantation was worse than that of the lower uterine implantation group. Through univariate analysis and logistic regression analysis, we found that the cervical width, abundant cervical blood flow, and bladder line interruption were all risk factors of PAS complicated with cervical implantation, and their contribution to the establishment of the regression model was statistically significant.

**Conclusion:**

PAS complicated with cervical implantation was extremely severe. Early identification of risk factors and establishment of a risk warning model have certain guiding significance for clinical formulation of a reasonable treatment plan.

## 1. Introduction

Placenta accreta spectrum (PAS), a serious obstetric disease, is characterized by the inability of placenta to be delivered by itself after delivery of fetus, and the tight adhesion between placenta and uterine wall during artificial placenta removal. Moreover, some adverse pregnancy outcomes, including severe obstetric bleeding, diffuse intravascular coagulation, and hysterectomy, may be induced once the villous tissue embedded in the myometrium is forcibly stripped [1, 2]. The incidence of PAS in most middle- and high-income countries has almost increased by 10 times, and that in the United States has increased by 10–15 times compared with 30–40 years ago in the context of increased Cesarean section rate and number of elderly pregnant women [1]. China is known to be among the highest Cesarean section rate all over the world. With the full liberalization of the “two-child” and “three-child” policies, the incidence of PAS is also rising rapidly, which is a tremendous problem faced by obstetrics in China.

Taking into account the high incidence and harmfulness of PAS, the academic community has conducted a lot of explorations on the classification of PAS, hemostasis methods, and perinatal management, which improves the pregnancy outcome of PAS patients to a certain extent. However, the PAS classification is still more based on the depth of the placental villi invading the myometrium, and there are still few reports about the lateral extension of the placenta, especially the reports of cervical involvement [3]. In 2019, we retrospectively analyzed 96 cases of PAS in our hospital and found that PAS patients with cervical implantation had more bleeding volume during Cesarean section and higher probability of hysterectomy and bladder injury than those with lower uterine implantation, which indicated that it was necessary to focus on the placenta implantation in cervix. However, due to the lack of clinical experience and professional knowledge of medical imaging, PAS complicated with cervical implantation is easy to be misjudged by obstetricians, leading to excessive surgery, even unnecessary hysterectomy, or delay in hysterectomy, resulting in the increase of risk. Therefore, there is an urgent need to establish a high-performance risk early warning model, which is bound to change this unhealthy situation.

Artificial intelligence (AI) is developing rapidly in many areas, such as the medical industry. In the research of obstetrics and gynecology, AI has been applied to fetal monitoring [4], prediction of premature delivery [5], prediction of postpartum hemorrhage risk [6], prediction of vaginal trial delivery after Cesarean section [7], and forceps midwifery [8]. The disease risk warning model, a statistical model based on big data, is an outstanding performance of artificial intelligence in the medical field. Clinicians are able to identify high-risk groups, improve medical decision-making, and ultimately improve patient prognosis using the risk warning model. The present study retrospectively analyzed the clinical and imaging data of 166 pregnant women with PAS in the Maternal and Child Health Hospital Affiliated to Nanchang University from 2016 to 2020, screened the risk factors of PAS patients complicated with cervical implantation, and established a disease risk early warning model, so as to guide clinicians to evaluate the condition accurately and formulate a reasonable surgical treatment plan.

## 2. Data and Methods

### 2.1. Study Population

The data of pregnant women with PAS who were hospitalized and delivered in the Maternal and Child Health Hospital Affiliated to Nanchang University from January 1, 2016, to September 30, 2020, were collected retrospectively. All medical records were retrieved through the medical record management system. The retrieval strategies were placental implantation as the discharge code and Cesarean delivery as the operation code. The inclusion criteria included singleton pregnancy and clinical description diagnosis or postoperative pathological biopsy diagnosis of placental implantation. The exclusion criteria included pregnant women with primary coagulation dysfunction or other serious pregnancy complications and pregnant women with incomplete medical records. Finally, a total of 166 pregnant women were included in this study. This study was approved by the hospital ethics committee.

### 2.2. Diagnostic Criteria

The diagnosis of PAS was based on surgical and/or pathological evidence. Specifically, it was defined as a large number of placental villi invading myometrium, serosa, and even organs outside the uterus. The diagnostic criteria for PAS complicated with cervical implantation were the presence of the placenta that is attached to the internal cervix during Cesarean section and could not be peeled off by itself. Meanwhile, the cervix was found to be incomplete during manual dissection or the postoperative tissue biopsy indicated the incompleteness of cervix or the presence of villous tissue. The diagnostic criteria of PAS complicated with lower uterine segment implantation were that the placenta could not be peeled off by itself during Cesarean section. Simultaneously, only the lower uterine segment was invaded, the cervical mucosa was smooth and intact, and the villus or myometrium was missing in the myometrium of the uterus by tissue biopsy.

### 2.3. Methods of Medical Imaging Examination

All patients were examined by two fixed and experienced ultrasound or imaging doctors within one week before the Cesarean section. The model of the ultrasonic diagnostic apparatus was GE Voluson E8, and the probe frequency was set as 5–9 MHz. The ultrasonic examination methods were as follows. The patient was asked to empty the bladder before examination, and abdominal color Doppler ultrasound was performed to check the growth diameter of the fetus, the attachment position of placenta, and the relationship between placenta and the internal cervix. Subsequently, the patient was instructed to take the bladder lithotomy position. After wrapping the vaginal ultrasound probe with sterile condom, the probe was inserted into the fornix vaginae and was gently rotated to the sagittal section of the maternal uterus for measuring the length of the cervix, the width of the cervix, the blood flow and shape of the cervix, and the bladder line. For PAS patients with obesity, posterior placenta, or controversial ultrasound diagnosis, pelvic MRI was additionally performed to assist in the diagnosis. The model of the MRI diagnostic apparatus was SIEMENS superconducting 1.5 T magnetic resonance instrument. And the MRI examination methods were as follows. PAS patients adopt left decubitus position, and multichannel body phased array coils were used to image the placenta and cervix in cross-section, coronal, and sagittal planes.

### 2.4. Cesarean Section

Two chief physicians with corresponding qualifications in placental disease ward would perform this surgery. The main points of the Cesarean section were as follows. (1) Abdominal aortic balloon implantation was performed before Cesarean section for the patients with highly suspected cervical implantation. (2) Epidural anesthesia was the main anesthesia method and general anesthesia under tracheal intubation would be applied if necessary. (3) Bladder was separated and pushed down to the level of the intrauterine mouth before the fetus was delivered. (4) The placenta should be avoided as much as possible when you choose the uterine incision; if the placenta could not be avoided, we should choose the place where the placenta was relatively thin. For patients with cervical implantation, the preset abdominal aortic balloon was filled at the same time as the fetus was delivered to block the blood supply of the uterus temporarily. (5) The uterus was dragged out and then the lower part of the uterus near the inner mouth was bundled up with the tourniquet. (6) When the placenta is implanted in the lower part of the cervix, we should strip out the placenta step by step with our hands and suture immediately. (7) The peeling surface of the placenta should be observed for about 15 minutes, and then the uterus was sutured if there was no active bleeding.

### 2.5. Estimation Method of Postpartum Bleeding Volume

According to the “Guidelines for Prevention and Treatment of Postpartum Hemorrhage” issued by the Obstetrics and Gynecology Committee of Chinese Medical Association, the volume of postpartum hemorrhage was evaluated by the combination of gauze weighing method and volumetric method. In the present study, negative pressure bottles and gauze were used to collect the bleeding during the perioperative period of emergency Cesarean section and the beginning of elective Cesarean section. The postoperative vaginal bleeding volume was calculated by the weighing method. The diagnostic criteria of postpartum hemorrhage, referring to the 2014 edition of clinical guidelines for diagnosis and treatment of postpartum hemorrhage, was that the bleeding volume within 24 hours after delivery was greater than 1000 ml.

### 2.6. Collection of Clinical Data

All clinical data was collected from our hospital's electronic medical record system, including basic information, the experience of the third trimester of pregnancy, imaging data, and delivery outcomes. The basic information included age, number of gravidities, times of induced abortions, and Cesarean sections. The third trimester of pregnancy mainly included the times of vaginal bleeding and the maximum volume of vaginal bleeding, and methods of volume and weighing were used to calculate the maximum vaginal bleeding volume. The imaging data included the attachment position of the main body of the placenta (anterior placenta or nonanterior placenta), the relationship between the placenta and the internal cervix (complete coverage or incomplete coverage), cervical length (distance between the internal and external cervical orifice), cervical width (left and right diameter of cervix), cervical blood flow (multiple anechoic areas of varying sizes in the cervix could be seen when cervical blood flow was abundant), cervical morphology, and bladder line (the high echo line between serosa and bladder cavity). The maternal outcome included gestational ages, postpartum bleeding volume, amount of blood transfusion, rate of hysterectomy, and bladder injury.

## 3. Statistical Analysis

IBM SPSS 24.0 software was used for data processing. The count data was expressed as frequency and rate, and the statistical analysis was performed with the chi-square test. The measurement data with a normal distribution was expressed as means and standard deviations, and the statistical analysis was performed using an independent sample *t* test. The measurement data with a skew distribution was expressed as median and quartile spacing, and the statistical analyses were performed using Mann–Whitney *U* test. Logistic regression was used to construct the risk prediction model of cervical implantation with PAS. ROC curve was used to evaluate the diagnostic ability of risk factors *f* cervical implantation with PAS. *P* < 0.05 was statistically significant.

## 4. Results

### 4.1. Distribution of Postpartum Bleeding Volume of the Two Groups

Among the 166 subjects, there were 49 cases of PAS complicated with cervical implantation and 117 cases of PAS complicated with lower uterine implantation. The postpartum hemorrhage rate of 68 patients with postpartum hemorrhage was 40.96% (68/166), of which the postpartum hemorrhage rate of cervical implantation group was 83.67% (41/49). The bleeding volume was mainly 1000 ml∼2000 ml, and the postpartum bleeding volume of 4 patients was as high as 3000 ml. The postpartum hemorrhage rate in the lower uterine implantation group was 23.08% (27/117), and the bleeding volume group was mainly 500 ml∼1000 ml. The chi-square test for trends showed that there was a linear trend between placental implantation position and postpartum bleeding volume. Details were shown in Table 1. The proportion of PAS complicated with cervical implantation increased with the increase of postpartum bleeding volume.

### 4.2. Maternal Outcomes in PAS Patients of the Two Groups

Comparing the maternal outcomes of PAS patients in the two groups, it was found that the amounts of bleeding volume, red blood cell transfusion, and plasma transfusion in Cesarean section in cervical implantation group were significantly higher than those in lower uterine implantation group. In addition, the hysterectomy rate and bladder injury rate in cervical implantation group were also significantly higher than those in lower uterine implantation group. See Table 2.

### 4.3. Univariate Analysis of PAS Complicated with Cervical Implantation

The independent sample *t* test, Mann-Whitney *U* test, and chi-square test were used to analyze the possible influencing factors of PAS complicated with cervical implantation. The results showed that the number of Cesarean sections, anterior placenta, complete placenta previa, bladder line interruption, cervical length, cervical width, abundant cervical blood flow, and cervical morphological disorder were all related to PAS complicated with cervical implantation. See Table 3.

### 4.4. Establishment and Validation of Logistic Regression Model for PAS Complicated with Cervical Implantation

The 8 independent variables obtained after univariate analysis were introduced into the logistic regression model, and the detailed results were shown in Table 4. The effects of eight variables in the prediction model were analyzed. The results showed that the cervical width (*X*_1_), abundant cervical blood flow (*X*_2_), and bladder line interruption (*X*_3_) contributed significantly to the regression model, which were independent risk factors of PAS complicated with cervical implantation, while the other five independent variables had little effect. Therefore, the prediction model was established as follows:

(1) $$\begin{array}{c} \overset{\wedge }{P}=\frac{exp\left(-16.584+0.352X_{1}+5.036X_{2}+2.514X_{3}\right)}{1+exp\left(-16.584+0.352X_{1}+5.036X_{2}+2.514X_{3}\right)}. \end{array}$$

The Hosmer–Lemeshow goodness-of-fit test showed 5.984 of *χ*^2^ and 0.649 of *P* valu*e*, indicating that the model had a good fit. The sensitivity of the prediction model was 91.84%, the specificity was 98.29%, the missed diagnosis rate was 8.16%, and the misdiagnosis rate was 1.71%.

### 4.5. Joint Diagnosis of PAS Complicated with Cervical Implantation by Multiple Independent Risk Factors

In this study, the logistic regression analysis showed that cervical width, abundant cervical blood flow, and bladder line interruption were independent risk factors of PAS with cervical implantation. When the cervical width was used as the diagnostic index alone, the optimal diagnostic threshold of cervical width was 33.5 mm and AUC was 0.854. When the abundant cervical blood flow and bladder line interruption were taken as diagnostic indexes, the corresponding AUC were 0.865 and 0.841, respectively. The joint diagnosis of these three independent risk factors showed 0.886 of AUC. Details were shown in Figure 1.

## 5. Discussion

Currently, the etiology of PAS remains controversial, and the mainstream etiology theory holds that its onset may be attributed to the secondary local tissue hypoxia during the process of uterine scar formation, resulting in abnormal vascularization, which further leads to the defect of uterine decidua and abnormal invasion of trophoblast cells into uterine myometrium and pelvic organs. The cervix, a special part of the uterus, is normally located in the deep position of the female pelvic cavity, mainly composed of connective tissue, with few smooth muscle fibers, blood vessels, and elastic fibers, and mainly receiving blood supply from the descending branch of uterine artery and part of vaginal artery. Once the placenta invades the cervix, the blood flow of the cervix increases, and the difficulties such as poor contraction of myometrium, wide bleeding wound, fast bleeding speed, and difficulty in stopping bleeding easily occur in the process of placental abruption [9], which seriously perplex the majority of obstetricians.

In 2020, Liu analyzed the clinical data of 105 cases of invasive placenta previa and found that 7 patients with cervical implantation had undergone hysterectomy due to severe bleeding [10]. In this study, 49 cases of PAS had cervical implantation, of which 41 cases had postpartum hemorrhage, 6 cases had hysterectomy due to intractable postpartum hemorrhage, and 6 cases had bladder injury due to placenta penetrating the cervix and invading the bladder. It was not unexpected to find out that the incidence of these three adverse outcomes in cervical implantation group was significantly higher than that in lower uterine implantation group by comparing the postpartum hemorrhage rate, hysterectomy rate, and bladder injury rate between cervical implantation group and lower uterine implantation group. As an obstetrician, it is of great clinical significance to determine whether PAS is complicated with cervical implantation before operation, so as to improve the safety of Cesarean section and improve the maternal outcome. Therefore, the early identification of the risk factors of PAS complicated with cervical implantation and the construction of a risk warning model are particularly essential.

Clinical indicators and medical imaging data are irreplaceable for obstetricians to assess the condition of PAS patients. The clinical indicators mainly include the patient's demographic characteristics, past medical history, and pregnancy history. The subjects included in this study were pregnant women with placenta previa complicated with placenta implantation. The clinical indicators included the clinical data of age, times of pregnancies, induced abortions, Cesarean sections, vaginal bleeding in the third trimester, and maximum volume of vaginal bleeding. Univariate analysis found that there was a correlation between the number of Cesarean sections and PAS complicated with cervical implantation, which was consistent with the current global PAS consensus, indicating that the incidence rate of PAS increased with the increase of Cesarean delivery [11–13]. Obstetricians are able to make a preliminary assessment of the disease through comprehensive analysis of various clinical indicators and decide on the supplementary examination that needs to be improved in the followup. At present, multimodal ultrasound imaging has been recommended by the diagnosis and treatment guidelines of PAS in various countries to accurately assess the high-risk women with PAS [14]. In the present study, color Doppler ultrasound was used as the preferred auxiliary examination, including transabdominal ultrasound and transvaginal ultrasound [15]. For patients with obesity or placenta in posterior wall, we performed pelvic MRI [16]. In addition to the common ultrasound signs of PAS, we paid special attention to cervix-related images in the included image data, including the length, width, blood flow, and morphology of the cervix. A univariate analysis of 7 imaging signs showed that these imaging signs were all related to PAS complicated with cervical implantation.

During the past years, the observation time window of cervical morphology was mainly in the second trimester of pregnancy which aimed to predict the incidence of preterm delivery. In recent years, based on the idea that changes of cervical morphology could reflect the changes of cervical load and surrounding structure, the observation indexes of cervical morphology have been gradually brought into the scope of imaging examination of placenta previa with placenta accrete. Polat et al. [9] thought that cervical shortening seemed to be a warning sign of placenta previa with penetration. Our study showed that the cervical length of PAS patients complicated with cervical implantation was significantly shorter than that of lower uterine implantation, which was consistent with Polat M's study. However, when the number of Cesarean sections and 7 imaging signs were used as independent variables for logistic regression analysis, the results showed that cervical width, abundant cervical blood flow, and bladder line interruption were independent risk factors of PAS complicated with cervical implantation. The optimal threshold value of cervical width was 33.5 mm. When other independent variables were fixed, the probability of cervical implantation in PAS increased by 0.421 times for every 1 mm increase in cervical width. When imaging examination showed abundant cervical blood flow, the probability of cervical implantation in PAS increased 152.851 times. In addition, the bladder is the organ closest to the lower part of the uterus and the cervix in the third trimester. The bladder line can reflect the relationship between bladder, lower part of the uterus, and cervix. If ultrasound or MRI indicates that the bladder line is interrupted, it means that the boundary between the bladder and the uterus is not clear. In this study, when the imaging examination showed that there was bladder line interruption, the probability of cervical implantation in PAS increased by 11.353 times. ROC analysis showed that the corresponding AUC were 0.854, 0.865, and 0.841, respectively, when cervical width, cervical blood flow, and bladder line interruption were used alone for diagnosis of PAS with cervical implantation. While the AUC was 0.886 when the three indexes were used for joint diagnosis, which indicated that the combined detection had good diagnostic value for PAS with cervical implantation.

There was no gainsaying the fact that, due to the nature of a retrospective single-center cohort study, the present study excluded some cases of missing data or insufficient imaging data, cases of twins, and pregnant women with multiple fetuses, which may have a certain impact on the results of the statistical analysis. Concurrently, the lack of data on the length and width of cervix in 166 patients with placental implantation before pregnancy or early pregnancy makes this study unable to accurately and dynamically evaluate the changes of cervix during pregnancy. More reliable models should be established with the help of the combined analysis of multicenter data in future researches.

## 6. Conclusion

PAS complicated with cervical implantation was extremely severe, which is often accompanied by adverse pregnancy outcomes such as postpartum hemorrhage, hysterectomy, and bladder injury. Preoperative image of Cesarean section has certain predictive value in predicting PAS with cervical implantation. Establishing the risk prediction model of PAS complicated with cervical implantation by logistic regression analysis before operation has positive significance in guiding obstetricians to formulate reasonable treatment plan.

## Figures and Tables

**Figure 1:** Risk prediction model and ROC curve of each risk factor.

**Table 1:** Distribution of postpartum bleeding volume of the two groups.

Postpartum bleeding volume (ml)	Cervical implantation group (case/rate)	Implantation group (case/rate)
<500 (*n* = 35)	2 (5.70%)	33 (94.30%)
500∼(*n* = 63)	6 (9.50%)	57 (90.50%)
1000∼(*n* = 48)	23 (47.90%)	25 (52.10%)
2000∼(*n* = 16)	14 (87.50%)	2 (12.50%
3000 (*n* = 4)	4 (100%)	0 (0)
Linear-by-linear association	57.047	
*P* value	<0.001	
Method	Monte Carlo	

**Table 2:** Maternal outcomes of the two groups.

	Cervical implantation group (*n* = 49)	Lower uterine implantation group (*n* = 117)	*P* value	Method
Bleeding volume (ml)	1800 (1000, 2100)	600 (400, 900)	<0.001	Mann-Whitney
Red blood cell transfusion (ml)	900 (500, 1450)	0 (0, 450)	<0.001	Mann-Whitney
Plasma transfusion (ml)	400 (0, 700)	0 (0, 100)	<0.001	Mann-Whitney
Hysterectomy (case/rate)	6 (12.25%)	0 (0)	0.001	Continuity correction
Bladder injury (case/rate)	6 (12.25%)	1 (0.86%)	0.001	Continuity correction

Data are presented as median (interquartile spacing).

**Table 3:** Univariate analysis of PAS complicated with cervical implantation.

	Cervical implantation group	Lower uterine implantation group	*P* value	Method
Age (years)	32 (30, 35)	30 (28, 34)	0.071	Mann–Whitney
Gravidity (times)	4 (3, 6)	4 (3, 5)	0.404	Mann–Whitney
Induced abortion (times)	1 (1, 3)	1 (1, 2)	0.790	Mann–Whitney
Cesarean section (times)	1 (1, 2)	1 (1, 2)	0.017	Mann–Whitney
Vaginal bleeding (times)	1 (0, 1.50)	1 (0, 2)	0.486	Mann–Whitney
Maximum volume of vaginal bleeding (ml)	10 (0, 90)	10 (0, 120)	0.767	Mann–Whitney
Anterior placenta (case/rate)	41 (83.70%)	64 (54.70%)	<0.001	Pearson
Complete placenta previa (case/rate)	48 (98%)	95 (81.20%)	0.004	Pearson
Cervical length (mm)	28.06 ± 6.37	33.67 ± 7.49	<0.001	Independent sample t
Cervical width (mm)	36.96 ± 6.22	28.25 ± 3.08	<0.001	Independent sample t
Abundant cervical blood flow (case/rate)	37 (75.50%)	3 (2.60%)	<0.001	Pearson
Morphological disorder of cervix (case/rate)	29 (59.20%)	5 (4.30%)	<0.001	Pearson
Bladder line interruption (case/rate)	38 (77.60%)	11 (9.40%)	<0.001	Pearson

Data are presented as median (interquartile spacing) or mean ± standard deviation.

**Table 4:** Logistic regression analysis of PAS complicated with cervical implantation.

	Β	SE	Wald	*P*	OR		95% CI
Cesarean section	−0.749	0.628	1.420	0.233	0.473		(0.138, 1.621)
Anterior placenta	−0.405	0.900	0.203	0.653	0.667		(0.114, 3.893)
Central placenta previa	−4.182	2.734	2.340	0.126	0.015		(0.000, 3.241)
Cervical length	−0.033	0.066	0.253	0.615	0.967		(0.851, 1.101)
Cervical width	0.352	0.111	9.987	0.002	1.421		(1.143, 1.767)
Abundant cervical blood flow	5.036	1.281	15.462	<0.001	153.851		(12.502, 1893.379)
Morphological disorder of cervix	1.472	0.970	2.303	0.129	4.356		(0.651, 29.136)
Bladder line interruption	2.514	0.940	7.151	0.007	12.353		(1.957, 77.976)
Constant	−16.584	5.423	9.352	0.002			

## Data Availability

The labeled dataset during the current study are available from the corresponding author on reasonable request.
